The article "Deep Transfer Learning for COVID-19 Detection and Lesion Recognition Using Chest CT Images" was published in 2022. Journal: Comput Math Methods Med.

# Deep Transfer Learning for COVID-19 Detection and Lesion Recognition Using Chest CT Images

**DOI:** 10.1155/2022/4509394

**Published:** 2022-10-15

**Authors:** Sai Zhang, Guo-Chang Yuan

**Affiliations:** ^1^Qualcomm Inc., 5775 Morehouse Drive, San Diego, CA 92121, USA; ^2^Department of Emergency Medicine, Union Hospital, Tongji Medical College, Huazhong University of Science and Technology, Wuhan 430022, China

## Abstract

Starting from December 2019, the global pandemic of coronavirus disease 2019 (COVID-19) is continuously expanding and has caused several millions of deaths worldwide. Fast and accurate diagnostic methods for COVID-19 detection play a vital role in containing the plague. Chest computed tomography (CT) is one of the most commonly used diagnosis methods. However, a complete CT-scan has hundreds of slices, and it is time-consuming for radiologists to check each slice to diagnose COVID-19. This study introduces a novel method for fast and automated COVID-19 diagnosis using the chest CT scans. The proposed models are based on the state-of-the-art deep convolutional neural network (CNN) architecture, and a 2D global max pooling (globalMaxPool2D) layer is used to improve the performance. We compare the proposed models to the existing state-of-the-art deep learning models such as CNN based models and vision transformer (ViT) models. Based off of metric such as area under curve (AUC), sensitivity, specificity, accuracy, and false discovery rate (FDR), experimental results show that the proposed models outperform the previous methods, and the best model achieves an area under curve of 0.9744 and accuracy 94.12% on our test datasets. It is also shown that the accuracy is improved by around 1% by using the 2D global max pooling layer. Moreover, a heatmap method to highlight the lesion area on COVID-19 chest CT images is introduced in the paper. This heatmap method is helpful for a radiologist to identify the abnormal pattern of COVID-19 on chest CT images. In addition, we also developed a freely accessible online simulation software for automated COVID-19 detection using CT images. The proposed deep learning models and software tool can be used by radiologist to diagnose COVID-19 more accurately and efficiently.

## 1. Introduction

In December 2019, unexplained illness attacked Wuhan, which was subsequently confirmed to be caused by a novel coronavirus called SARS-CoV-2, and the infection caused by it was named COVID-19. The World Health Organization (WHO) declared the new type of coronavirus infection as a Public Health Emergency of International Concern (PHEIC) on January 31, 2020. The cumulative number of COVID-19 infections worldwide has exceeded 110 million, and the death toll has stood over 2.6 million [1].

The article "Deep Transfer Learning for COVID-19 Detection and Lesion Recognition Using Chest CT Images" was published in 2022. Journal: Comput Math Methods Med.

COVID-19 has many similarities with common respiratory viral infections. The main clinical manifestations are dry cough, fever, fatigue, and dyspnea. Some cases may have a sore throat, chest pain, myalgia, and diarrhea [2, 3]. Severe cases may rapidly develop into acute respiratory distress syndrome (ARDS), sepsis, and renal failure [4]. The “Next-Generation” sequencing (NGS) and reverse transcription-polymerase chain reaction (RT-PCR) test are the most commonly used methods for COVID-19 detection. However, NGS and RT-PCR tests are accurate only when properly performed by health care professionals. The rapid COVID tests and self-tests can miss some cases. The inadequate sensitivity of the RT-PCR test may result in false negatives and more potential infections [5]. The research in [6] showed that the joint detection of nucleic acid and antibodies could increase the true positive rate of COVID-19. The study in [7] found that among 1014 suspected cases, the positive rate of RT-PCR test and lung CT was 59% and 88%, respectively, indicating that lung CT has a higher sensitivity to COVID-19. In [8], it is shown that for suspected cases with a negative nucleic acid test, chest CT examination is necessary to improve the accuracy of diagnosis. The main chest CT manifestations of COVID-19 are bilateral, peripheral/subpleural, posterior ground-glass opacity, crazy paving pattern, and consolidation. Some patients may have air bronchogram, bronchial wall thickening, lung nodules, pleural effusion, pleural thickening, lymphadenopathy, and other abnormalities [9–11].

At present, image processing, computer vision, and artificial intelligence (AI) have been extensively used in medical imaging and digital health applications [12–18] due to their excellent performance on image classification and target detection [19, 20]. These techniques are used in various medical diagnostic applications such as lung nodules classification based on CT images [21], heart rhythm monitoring [22], brain tumor classification from MRI images [23], and breast cancer detection using histopathology images [24]. These methods can help physicians speed up the analysis, arrive at a more accurate diagnosis, and develop appropriate treatment.

The motivation of this study is to design a fast, accurate, and automated method for COVID-19 detection using the CT scans. Fast diagnostic method can curb and control the spread of COVID-19. In this paper, several deep transfer learning models for COVID-19 detection based on chest CT images are proposed. The proposed models can be used as a supplement or alternative to the RT-PCR test in high incidence areas for faster and more accurate COVID-19 diagnosis.

The article "Deep Transfer Learning for COVID-19 Detection and Lesion Recognition Using Chest CT Images" was published in 2022. Journal: Comput Math Methods Med.

The contributions of this paper are summarized as follows in bullet points:

- A large and specialist verified dataset is used for training, validation, and testing. The dataset was collected from Wuhan Red Cross Hospital during the pandemic from January to March 2020. A large and practical dataset is crucial in machine learning
- Convolutional neural network architectures such as VGG19 and ResNet50V2 are used for COVID-19 detection based on CT images. In addition, we proposed an improvement to use the 2D global max pooling layer instead of the commonly used flatten layer or 2D global average pooling layer to help feature extractions. Experimental results show that the accuracy is improved by around 1% by using the 2D global max pooling, and the VGG19 model with the 2D global max pooling layer has the best performance
- Additionally, we compare the proposed models to the state-of-the-art models in the literature, including ViT, MobileNetV2, InceptionResNetV2, and ResNet152V2. The proposed VGG19+MaxPool2D model outperforms the previous methods and can achieve an accuracy rate of 94.12%.
- We introduce a heatmap method to highlight the lesion area on the COVID-19 chest CT images. Results show that a clear heatmap on the lesion area can be obtained using the proposed models. This heatmap method is helpful for a radiologist to identify the abnormal pattern of COVID-19 on chest CT images faster. Compared to the existing literature such as [25], the proposed transfer learning based models achieve a better accuracy and more reasonable lesion area heatmap
- We developed a freely accessible online software for COVID-19 detection and lesion area localization using CT image. Using this software requires no programming or machine learning background. The proposed models and software tool can be used to accelerate and improve the accuracy of diagnosis of COVID-19, which can help control the pandemic

The rest of the paper is organized as follows. The related works on COVID-19 detection using AI is presented in Section 2. In Section 3, the datasets used in this study are introduced.  Section 4 describes the proposed deep learning models. The training and validating process of all models are also described in Section 4. In Section 5, experimental results (inference results on the test dataset) for all proposed models are presented. Comparison between the proposed models and the other state-of-the-art techniques is also given.  Section 6 introduces a heatmap method to visualize the abnormal pattern in the COVID-19 CT images. In Section 7, we describe a newly developed online software for COVID-19 detection. Finally, concluding remarks are given in Section 8.

The article "Deep Transfer Learning for COVID-19 Detection and Lesion Recognition Using Chest CT Images" was published in 2022. Journal: Comput Math Methods Med.

## 2. Related Works and Background

The AI-based COVID-19 detection has become a hot spot and has attracted many researchers recently. A comprehensive review of AI-based COVID-19 detection literature was provided in [26]. In [27], the authors compared ten traditional convolutional neural networks to distinguish COVID-19 from non-COVID-19: AlexNet, VGG-16, VGG-19, SqueezeNet, GoogleNet, MobileNet-V2, ResNet-18, ResNet-50, ResNet-101, and Xception. Among these models, ResNet-101 performed the best and could identify COVID-19 with an AUC of 0.994. However, a comparatively small dataset with 1020 CT slices is used. Hence, a larger dataset is needed to validate their results. The authors in [28] proposed integrating chest CT findings with clinical history of patients for diagnosing COVID-19. In this study, a CNN is used for CT image-based diagnosis, and a multilayer perceptron (MLP) is used to classify COVID-19 based on the clinical history. By combining the CNN and MLP results, the authors state that the proposed algorithm achieves an AUC of 0.92. In [29], the authors developed a deep learning classifier based on ResNet50. The designed model could distinguish COVID-19 from other lung pathologies, such as lobar bacterial pneumonia, atypical or viral pneumonia, lung cancer, and infectious bronchiolitis, and achieved an AUC of 0.956 on an independent testing dataset. Similarly, a new multiclassification deep learning model was proposed for diagnosing COVID-19, pneumonia, and lung cancer chest diseases [30]. Four architectures were considered in this paper: VGG19, ResNet152V2, ResNet152V2+Gated Recurrent Unit (GRU), and ResNet152V2+Bidirectional GRU (Bi-GRU). The authors found that VGG19 performed the best and achieved 98.05% accuracy. An efficient deep learning technique to detect COVID-19 patterns in chest CT images named EfficientCovidNet is proposed in [31] for COVID-19 classification using CT images. The limitation in [29–31] is that it does not analyze an entire 3D dataset of DICOM images since the open-source data only contains the slices with pathological alterations of the lungs. More diverse datasets are needed to evaluate these techniques.

The researchers in [32] implemented the DenseNet201 model with transfer learning for COVID-19 detection based on chest CT images. The proposed model achieves an accuracy of 96.25% on their test dataset. In [33], the authors proposed a computer-aided diagnosis (CAD) system to detect COVID-19 based on several methods, including deep end-to-end learning, deep feature extraction, and principal component selection. In [25], the authors proposed a two steps COVID-19 classification using a 3D CT volume. Firstly, the ResNet50 model is used to classify each CT image, and then, an AI method fuses image-level predictions to diagnose COVID-19 on a 3D CT volume. All works mentioned above have reasonable accuracy for COVID-19 classification. However, these models only output classification results (COVID-19 or non-COVID-19), but do not provide any information on the lesion area or the abnormal pattern in the CT images.

The article "Deep Transfer Learning for COVID-19 Detection and Lesion Recognition Using Chest CT Images" was published in 2022. Journal: Comput Math Methods Med.

In [34], a light CNN model based on the SqueezeNet was introduced for distinguishing COVID-19 from other community-acquired pneumonia or healthy cases. The class activation mapping (CAM) method is used to understand the behavior of the CNN models. It is shown in the paper that most of the activation is localized on the lesion part of the lung CT image. Compared to [25], the proposed models in our work provide a more accurate COVID-19 detection results and more reasonable lesion area localization results due to more complicated models, transfer learning, and a larger dataset.

There are also some studies focused on the impact of COVID-19. The researchers in [35] implemented a machine learning technique for predicting the death and cure rates of patients. In [36], an analysis of socioeconomic impacts of COVID-19 on public health is presented. Machine learning and data mining strategies are used in the analysis.

More details of related studies are provided in Table 1.

## 3. Datasets for the Study

We retrospectively collected 768 chest CT images (160639 CT slices) from 309 patients, including 20 patients without lung disease and 289 patients with COVID-19. The CT images are collected in Wuhan Red Cross Hospital from January to March 2020, and each chest CT image consists of 300 slices approximately. The CT slices are originally in DICOM format, and we converted them to JPG format with size 224^∗^224 pixels using the software Miele-LXIV. All slices were reviewed by senior respiratory specialists in Wuhan Union Hospital and labeled as three classes: non-COVID-19, COVID-19, or unclear (cannot be used to decide COVID-19). In this paper, we formulate the COVID-19 detection problem as a binary classification problem. Therefore, only slices that are labeled as non-COVID-19 and COVID-19 are used. Examples of the CT slices in the datasets are shown in Figure 1: Figures 1(a)–1(d) are examples of CT slides from COVID-19 patients, and Figures 1(e)–1(f) are examples of CT slides from non-COVID-19 patients.

The CT slices are split into training, validation, and test datasets. The 148,129 CT slices from the first 280 patients are randomly split into training and validation dataset, with the ratio of number of slices to be 4 : 1. The training set contains 118,506 slices (including 38,938 slices in non-COVID-19 and 79,568 slices in COVID-19). The validation set contains 29,623 slices (including 7,933 slices in non-COVID-19 and 19,890 slices in COVID-19). The rest of the 12,510 slices from 29 patients are used as test sets (including 6,136 slices in non-COVID-19 and 6,374 slices in COVID-19). Note that the slices in the test dataset are never seen by the model during training and validating process, since they are from different patients. Therefore, the inference results on the test dataset is an unbiased estimate of the skill of the trained model.

The article "Deep Transfer Learning for COVID-19 Detection and Lesion Recognition Using Chest CT Images" was published in 2022. Journal: Comput Math Methods Med.

## 4. Proposed Deep Learning Models for COVID-19 Detection

### 4.1. Proposed Models

The convolutional neural network (CNN) architecture is popular in computer vision and image classification problems due to its particular convolutional layer [37–41]. The main advantage of using convolutional layers is its high-level feature extraction ability in images.

In this study, we investigated the VGG19 and ResNet50V2 CNN architectures. The aim is to explore their performance in COVID-19 diagnosis using CT scans. We also proposed using a 2D global max pooling layer instead of the commonly used flatten layer or 2D global average pooling layer to improve the performance. Additionally, we compare the proposed models with the other existing state-of-the-art techniques such as Vision Transformer, MobileNet, InceptionResNetV2, and ResNet152V2. Details of the deep learning models used in this study are provided below.

#### 4.1.1. VGG19 CNN Models

The VGG19 architecture is a widely used deep sequential CNN model. In our work, we use the transfer learning method, and the pretrained convolutional layers of VGG19 architecture are used. The ImageNet weights are used to initialize the weights of the convolutional layers. Note that using the pretrained convolutional layers is a practical and common approach for improving the performance in deep learning problems [41, 42].

At the end of the convolutional layers, a flatten layer, a dense layer, a dropout layer, and a densely connected classifier are appended. We use a block diagram to conclude the structure of the proposed VGG19 based models as in Figure 2. In the state-of-the-art VGG19 architecture, the flatten layer is used to convert the output (with dimension 7 × 7 × 512) of the last convolutional layer and maxPoolingLayer to 1-dimensional linear vector (dimension 1 × 25088). In this study, a 2D global average pooling layer or a 2D global max pooling layer is used as an alternative to the flatten layer. The 2D global average/max pooling layer is used to average/max all the values in the pooled feature map after the last convolutional layer and max pooling layer.  Figure 3 is a visual representation of what this process looks like. Experimental results in Section 5 show that using 2D global max pooling can improve the performance for COVID-19 detection. More details about the VGG19 architecture can be found in [41, 42].

The article "Deep Transfer Learning for COVID-19 Detection and Lesion Recognition Using Chest CT Images" was published in 2022. Journal: Comput Math Methods Med.

#### 4.1.2. ResNet50V2 CNN Models

The ResNet model initially proposed in [43] utilized the residual learning framework. The residual learning framework helps in resolving the gradient vanishing problem in deep CNN. In our ResNet50V2 based CNN model, the pretrained convolutional layers of ResNet50V2 architecture are used. The ImageNet weights are used to initialize the convolutional layers.

Similar to the proposed VGG19 based models, the output of the last convolutional layer of ResNet50V2 is passed to the flatten layer, 2D global average pooling layer, or 2D global max pooling layer. Finally, a dense layer, a dropout layer, and a densely connected classifier are appended. The architecture of the ResNet50V2 based models is presented in Figure 4.

More details about the ResNet architecture can be found in [43].

#### 4.1.3. Other State-of-the-Art Deep Learning Models

In this study, we compared the proposed VGG19 and ResNet based models to several state-of-the-art deep learning models: Vision Transformer (ViT), MobileNetV2, InceptionResNetV2, and ResNet152V2.

The ViT model is based on the architecture of transformer originally designed for text or natural language processing. The researchers in [39] show that by dividing images into patches, the transformer can be applied to sequences of image patches for image classification tasks. It is shown that ViT attains excellent results compared to the state-of-the-art CNN when the training dataset is large. The detail architecture of the multihead attention, and ViT can be found in [39].

MobileNetV2 is a light-weight deep CNN architecture with 52 convolutional layers and 1 fully connected layer. The new depthwise separable convolution is used to reduce the weight in the architecture. MobileNetV2 has advantages such as faster computation and lower latency; therefore, it is used widely in mobile applications. More details about the MobileNet architecture can be found in [44].

InceptionResNetV2 is a deep CNN architecture with 164 layers. It is based on the Inception architecture and incorporates the residual connections from ResNet. The Inception part performs multiple convolutions on the same level with different filter sizes to reduce computational costs. The ResNet part utilizes the residual learning framework to help resolving the gradient vanishing problem. More details about the InceptionResNet architecture can be found in [45].

The article "Deep Transfer Learning for COVID-19 Detection and Lesion Recognition Using Chest CT Images" was published in 2022. Journal: Comput Math Methods Med.

ResNet152V2 is similar to ResNet50V2 but has different residual blocks scheme and different number of residual blocks. More details about the ResNet152V2 architecture can be found in [43].

### 4.2. Training of the Proposed Models

The general procedure of the training process is given in Algorithm 1. The preprocessing in Algorithm 1 step 2 includes data normalization and data augmentation. The data normalization is applied to both training and validation data. The normalization consists of two steps: (1) resize all the images to standard size using the basic bilinear interpolation image resizing method: 224 pixels height and 224 pixels width. Resizing is needed to keep up the computation limitations. (2) Normalize the value of each pixel in the image based on the model requirements: for the VGG19 and ViT models, the normalized value is between 0 and 1. For the ResNet, MobileNet, and InceptionResNet models, the pixel value is normalized to between -1 and 1.

The data augmentation preprocessing is applied only to the training datasets. Data augmentation is a technique used to increase the amount of data by applying random transformation on existing CT images to create slightly modified copies. It is a commonly used method to solve the overfitting problem during the training, especially when the dataset is small. In our study, the following random transformation is applied: (1) randomly rotate the image from -40 to 40 degrees; (2) randomly shift the image horizontally (left or right) by 0 to 8 pixels; (3) randomly shift the image vertically by 0 to 15 pixels (up and down); and (4) randomly apply shearing transformation from 100% (no shearing) to 110%. Note that shearing is to distort the image along the *x* or *y* axis to create the perception angles; (5) randomly zooming the image from 100% (no zooming) to 110%; and (6) randomly flip the image horizontally or/and vertically. Some examples of the augmented images are shown in Figure 5: An example of the original CT slice that labeled as COVID-19 is shown in Figure 5(a). Examples of augmented CT slice such as vertically flipped, rotated, and shifted in horizontal direction are shown in Figures 5(b)–5(d), respectively.

After preprocessing, we train the model using the training dataset. Each iteration of the training process is called an epoch. The number of epochs is set to 100 in this study. Since the COVID-19 detection is formulated as a binary classification problem, we use the binary cross-entropy function as the loss function for weight update during the training process. The binary cross-entropy loss function is defined in

(1) $$\begin{array}{c} \text{Loss}\left(y\right)=-\frac{1}{N}\overset{N}{\underset{i=1}{\sum }}y_{i}\log\left(p\left(y_{i}\right)\right)+\left(1-y_{i}\right)\log\left(1-p\left(y_{i}\right)\right), \end{array}$$

where **y** = [*y*_1_*y*_2_*y*_3_, ⋯, *y*_*i*_], and *y*_*i*_ is the label for the *i*^th^ image (label 1 for COVID-19 and label 0 for non-COVID-19), and *p*(*y*_*i*_) is the predicted probability of the *i*^th^ image being COVID-19. Since the model is doing binary classification, the accuracy of the model is defined as the percentage of the predicted values that match with the actual values for the binary labels.

The article "Deep Transfer Learning for COVID-19 Detection and Lesion Recognition Using Chest CT Images" was published in 2022. Journal: Comput Math Methods Med.

The flowchart of the overall COVID-19 recognition system design is presented in Figure 6. Other parameters of the system and the simulation environment are given below:

1. The batch size is set to 32 in the training and validating process. The number of steps per epoch is calculated to be the total number of images divided by the batch size
2. Transfer learning is used to optimize the deep learning models. The ImageNet weights are used to initialize the weights in the convolutional layers in all CNN models. For the ViT model, the multihead attention layers are initialized by the ImageNet weights
3. For all models, the binary cross-entropy function mentioned in Equation (1) is used as the loss function, and we use the Adam optimizer to update the weights of the models. The initial learning rate is set to 1e-4
4. When training the CNN models, we first freeze the weights in the convolutional layers and only trained the dense layers for 5 epochs. This is to ensure that the pretrained ImageNet weights in the convolutional layers will be not messed up by the randomly initialized weights in the dense layer. Then, the convolutional layers are jointly trained with the base layers for 95 epochs
5. When training the ViT model, we first freeze the weights in the multihead attention blocks and only trained the dense layer for 5 epochs. Then, all the layers are jointly trained for 95 epochs
6. The training, validating, and testing process are performed using a Windows 10 desktop with an NVIDIA GeForce RTX 2060 Graphic card. For the CNN models, the simulation is performed in Python 3.6 environment with tensorflow 2.1.0. For the ViT, the simulation is performed in Python 3.8 environment with tensoflow 2.8.0

### 4.3. Results of Training and Validation

The training and validating process of the proposed VGG19 based models are indicated in Figures 7(a)–7(c). It is shown that the VGG19 with flatten layer, VGG19 with 2D global average pooling layer and VGG19 with 2D global max pooling layer achieve training accuracy of 99.60%, 99.61%, and 99.64%, respectively. And the validation accuracy for the proposed VGG19 based models is 98.45%, 98.69%, and 99.07%, respectively.

The article "Deep Transfer Learning for COVID-19 Detection and Lesion Recognition Using Chest CT Images" was published in 2022. Journal: Comput Math Methods Med.

The training and validating process of the proposed ResNetV2 based models are presented in Figures 7(d)–7(f). The proposed ResNet50V2 with flatten layer, ResNetV2 with 2D global average pooling layer, and ResNet50V2 with 2D global max pooling layer achieve training accuracy of 99.70%, 99.83%, and 99.70, respectively. And the validation accuracy for the proposed ResNet50V2 based models is 98.89%, 98.67%, and 98.88%, respectively.

The training and validation process of the state-of-the-art benchmarking models are indicated in Figures 7(g)–7(j). The ViT, MobileNetV2, InceptionResNetV2, and ResNet152V2 achieve training accuracy of 87.06%, 99.74%, 99.91%, and 99.79%, respectively. And the validation accuracy for the four benchmarking models is 88.42%, 96.15%, 98.84%, and 97.55%, respectively.

The training time and number of parameters for all models are indicated in Table 2. Note that using a 2D global average/max pooling layer instead of the flatten layer can decrease the number of learning parameters in the model.

## 5. Experimental Results

The classification performance of the proposed models is evaluated on the test dataset. Note that the performance on the test data set will be the performance of the models on the CT images it has never seen before. Therefore, it is an unbiased performance measure of the proposed models.

For each model, the following performance metrics are calculated based on the inference results on the test dataset: sensitivity, specificity, accuracy, false discovery rate (FDR), and area under curve (AUC). The metrics and terms in the equations are defined as follows:

- Sensitivity: Sensitivity is the ability of the model to correctly identify the patients with a COVID-19. It is mathematically defined as in Equation (2)
- Specificity: Specificity is the ability of the model to correctly identify the people without COVID-19. It is mathematically defined as in Equation (3).
- Accuracy: Accuracy is the ability of the model to make a correct decision on whether the people are with COVID-19 or non-COVID-19. It is mathematically defined as in Equation (4).
- False discovery rate (FDR): FDR is the ratio of the number of false positive (COVID-19) results to the number of total positive results. It is mathematically defined as in Equation (5).
- Area under curve: The area under the ROC curve measures the usefulness of the model. In general, a greater area under the curve means a more valuable and accurate model

(2) $$\begin{array}{c} Sensitivity=\frac{\text{TP}}{\text{TP}+\text{FN}}, \end{array}$$

(3) $$\begin{array}{c} Specificity=\frac{\text{TN}}{\text{TN}+\text{FP}}, \end{array}$$

(4) $$\begin{array}{c} Accuracy=\frac{\text{TP}+\text{TN}}{\text{TP}+\text{TN}+\text{FP}+\text{FN}}, \end{array}$$

(5) $$\begin{array}{c} FDR=\frac{\text{FP}}{\text{TP}+\text{FP}}, \end{array}$$

where the TP (number of true positive), TN (number of true negative), FP (number of false positive), and FN (number of false negative) in Equations (2)–(5) are defined as below in bullet points [46]:

- TP (number of true positive): An output is called true positive when the model recognizes the CT image as positive (COVID-19), and the actual CT image is positive. The total number of images that are true positive is defined as TP
- TN (number of true negative): An output is called true negative when the model recognizes the CT image as negative (non-COVID-19), and the actual CT image is negative. The total number of images that are true negative is defined as TN
- FP (number of false positive): An output is called false positive when the model recognizes the CT image as positive, and the actual CT image is negative. The total number of images that are false positive is defined as FP
- FN (number of false negative): An output is called false negative when the model recognizes the CT image as negative, and the actual CT image is positive. The total number of images that are false negative is defined as FN

Figure 8 represents ROC curves for all proposed models and state-of-the-art benchmarking models. It is shown that the proposed VGG19 with 2D global max pooling layer model has the best ROC performance and achieves an AUC of 0.97744. We can also see that the proposed VGG19 with 2D global max pooling outperforms the state-of-the-art models such as ViT, MobileNetV2, InceptionResNetV2, and ResNet152V2. By comparing the AUC among the proposed VGG19 (or ResNet50V2) with flatten layer, VGG19 with 2D global average pooling layer, and VGG19 with 2D global max pooling layer, it is shown that using 2D global max pooling layer has the largest AUC. Besides, we use Youden's index to obtain the thresholds and evaluate the confusion matrix, sensitivity, specificity, accuracy, and FDR for all models on the test dataset. A confusion matrix is a table that contains TN, FP, FN, and TP values and is used to describe the performance of a classification model. The confusion matrix results are presented in Figures 9(a)–9(j), and Table 3 indicates the diagnostic performance of all models. Observations from Table 3 are concluded as below:

1. The proposed three VGG19 based models could distinguish COVID-19 from non-COVID-19 with accuracy 93.29%-94.12%. The proposed three ResNet50V2 based models achieve accuracy 91.85%-93.96%
2. The best accuracy performance was achieved by VGG19 with 2D global max pooling with accuracy 94.12%, and it outperforms the benchmarking models (ViT, MobileNetV2, InceptionResNetV2, and ResNet152V2 with accuracy 80.02%, 90.38%, 93.13%, and 90.78%, respectively)
3. By comparing the performance among VGG19 (or ResNet50V2) with flatten layer, VGG19 with 2D global average pooling layer, and VGG19 with 2D global max pooling, we found that using 2D global max pooling layer improves the accuracy by around 1%
4. The best sensitivity performance is achieved by VGG19 and ResNet50V2 with 2D global max pooling layer (with specificity 91.40% and 91.54%, respectively). The best specificity is achieved by VGG19 with 2D global max pooling and ResNet50V2 with 2D global average pooling (with specificity 96.95% and 97.51%, respectively). The best FDR is achieved by VGG19 with 2D global max pooling and ResNet50V2 with 2D global average pooling (with FDR 3.11% and 2.67%, respectively).

The article "Deep Transfer Learning for COVID-19 Detection and Lesion Recognition Using Chest CT Images" was published in 2022. Journal: Comput Math Methods Med.

Note that running the prediction on the test set (including 12510 CT slices) to label the CT slices only takes around 80 to 120 seconds. Therefore, these fast predictions can be used to accelerate the diagnosis of COVID-19.

## 6. Visualizing the Abnormal Pattern

This study also introduces a heatmap method to visualize the abnormal pattern in the COVID-19 CT image. The method is based on the class activation map (CAM) visualization techniques: a score of how vital each pixel is for classification is computed using a gradient method [47]. A heatmap image can be generated from the scores to indicate each pixel's importance for the abnormal pattern. The generated heatmap results for our proposed CNN models are shown in Figure 10. The highlighted region indicates a higher possibility for an abnormal pattern such as ground-glass opacity, crazy paving pattern, and consolidation. The abnormal pattern visualization heatmap results can be helpful for radiologist to identify the COVID-19 using CT image more accurately and efficiently.

## 7. Online Software for COVID-19 Detection

In order to present the developed COVID-19 classification models and make them helpful in assisting COVID-19 detection, we also developed a freely accessible online simulation software for COVID-19 detection. The proposed VGG19 with 2D global max pooling model is used in the software. Classification of a new CT image in the software can be performed by click on the “Choose File” button to select the CT image and then click on the “Recognize Image” button to generate output. As a result, using the software requires no programming and machine learning experience. The intuitive interface allows for COVID-19 detection and visualization of abnormal patterns in the CT image, as shown in Figure 11.

The article "Deep Transfer Learning for COVID-19 Detection and Lesion Recognition Using Chest CT Images" was published in 2022. Journal: Comput Math Methods Med.

Note that the online software is currently running on our own desktop server. Please email us to get the link to the software if interested.

## 8. Conclusion

In this paper, several deep learning models are designed and evaluated for fast and automated COVID-19 diagnosis using the chest CT scans. Six architectures are presented in this study: VGG19 with flatten layer, VGG19 with 2D global average pooling layer, VGG19 with 2D global max pooling layer, ResNet50V2 with flatten layer, ResNet50V2 with 2D global average pooling layer, and ResNetV2 with 2D global max pooling layer. We showed that by using the 2D global max pooling layer instead of the flatten layer or 2D global average pooling layer, we can improve the accuracy for COVID-19 detection by around 1%. Through extensive experiments performed on the test dataset, the VGG19 with 2D global max pooling layer model outperforms other proposed models and achieved 94.12% accuracy, 91.40% sensitivity, 96.95% specificity, 3.11% FDR, and 0.9744 AUC. We also compare the proposed model with various existing state-of-the-art techniques, such as ViT, MobileNet, InceptionResNetV2, and ResNet152V2 on the test dataset, and found superior diagnostic accuracy.

Moreover, we introduced a heatmap method to highlight the lesion area of the COVID-19 chest CT images, which helps identify the abnormal pattern in COVID-19 chest CT images. We also developed a freely accessible online simulation software for COVID-19 detection using CT images. The proposed method and software can accelerate the radiology checking process, and the classification speed can be as quick as 1.1 ms per CT image. It is important to efficiently and correctly diagnose the disease early to help control the epidemic.

## Figures and Tables

**Figure 1:** Examples of COVID-19 and non-COVID-19 CT images. (a–d) A 76-year-old male with confirmed COVID-19. (e–f) A 31-year-old female with non-COVID-19.

**Figure 2:** Structure of VGG19 based model.

**Figure 3:** Process of 2D global average or max pooling.

**Figure 4:** Structure of ResNet50V2 based model.

**Figure 5:** Examples of the augmented images. (a) original image; (b) flipped image; (c) randomly rotated image; and (d) randomly shifted image.

**Figure 6:** Flowchart of COVID-19 recognition system design.

**Figure 7:** Accuracy and loss plot of all models for training and validation datasets.

**Figure 8:** Receiver operating characteristic for all models (evaluated on the test datasets).

**Figure 9:** Confusion matrix of all models.

**Figure 10:** Heatmap and lesion area recognition for proposed models.

**Figure 11:** Online software for COVID-19 detection and pattern recognition.

The article "Deep Transfer Learning for COVID-19 Detection and Lesion Recognition Using Chest CT Images" was published in 2022. Journal: Comput Math Methods Med.

**Algorithm 1:** Train the proposed models.

**Table 1:** Summary of related work on deep learning based COVID-19 detection.

Ref.	Class	Subjects	Models	Sens. (%)	Spec. (%)	Prec. (%)	Acc. (%)	AUC (%)
Ardakani, Kanafi et al. [27]	COVID-19/other pneu.	108/86	ResNet-101	100.00	99.02	N/A	99.51	99.40
Mei, Lee et al. [28]	COVID-19/non-COVID-19	419/486	ResNet-18	84.30	82.80	N/A	N/A	92.00
Javor, Kaplan et al. [29]	COVID-19/other pneu.	209/209	ResNet-50	84.40	93.70	N/A	N/A	95.60
Silva, Luz et al. [31]	COVID-19/non-COVID-19	276/115	EfficientCovidNet	N/A	N/A	N/A	87.68	90.15
Jaiswal, Gianchandani et al. [32]	COVID-19/non-COVID-19	1263/1230	DenseNet201	N/A	96.21	96.29	96.25	97.00
Attallah, Ragab et al. [33]	COVID-19/non-COVID-19	347/397	Other CNN	95.90	93.70	N/A	94.70	98.00
Polsinelli, Cinque et al. [25]	COVID-19/non-COVID-19	460/397	Other CNN	87.55	81.95	85.01	85.03	N/A

**Table 2:** Characteristic of the models used in the study.

	Parameters (10^6^)	Training time per epoch (second)
VGG19 with flatten layer	32.87	1707
VGG19 2D globalAvgPooling	20.29	1704
VGG19 2D globalMaxPooling	20.29	1690
ResNet50V2 with flatten layer	74.95	1446
ResNet50V2 2D globalAvgPooling	24.61	1449
ResNet50V2 2D globalMaxPooling	24.61	1440
ViT	87.85	1863
MobileNetV2	2.26	1454
InceptionResnetV2	55.12	2080
ResNet152V2	59.38	2543

**Table 3:** Diagnostic performance for the deep learning models.

	AUC	Sensitivity	Specificity	Accuracy	FDR
VGG19 with flatten layer	0.974	90.97%	96.05%	93.46%	4.01%
VGG19 2D globalAvgPooling	0.976	91.18%	95.49%	93.29%	4.55%
VGG19 2D globalMaxPooling	0.977	91.40%	96.95%	94.12%	3.11%
ResNet50V2 with flatten layer	0.955	88.01%	95.84%	91.85%	4.35%
ResNet50V2 2D globalAvgPooling	0.963	87.67%	97.51%	92.49%	2.67%
ResNet50V2 2D globalMaxPooling	0.973	91.54%	96.48%	93.96%	3.57%
ViT	0.872	74.02%	86.25%	80.02%	15.17%
MobileNetV2	0.957	89.54%	91.26%	90.38%	9.66%
InceptionResnetV2	0.969	90.19%	96.19%	93.13%	3.91%
ResNet152V2	0.947	87.17%	94.54%	90.78%	5.69%

## Data Availability

The data that support the findings of this study are available from the corresponding author upon request.
